RETRACTED

# Analysis of Color Language and Aesthetic Paradigm of Print Art Based on GB-BP Neural Network

**DOI:** 10.1155/2021/4383092

**Published:** 2021-08-12

**Authors:** Zhiqiang Chen, Yongding Tan

**Affiliations:** College of Fine Arts and Design, Lingnan Normal University, Zhanjiang, Guangdong 524048, China

## Abstract

Color is the basic element of printmaking art creation and also an important medium for artists to express their emotions. In order to improve the understanding of the print by tourists, the research first carries out image analysis of different colors, summarizes the common color image adjectives in the art of publishing and painting, then optimizes BP neural network algorithm by gradient promotion (GP) algorithm, and constructs a color language analysis technology based on GP-BP neural network review paradigm. Through this technology, the content of color expression of different types of print art works is analyzed. Then, the subjective evaluation of these print art works is carried out by questionnaire adjustment method. Finally, the subjective evaluation and network evaluation results are compared. On the three materials, the expression effect of color image adjectives such as “heavy light fast,” “modern classical,” “lively steady,” and “soft Yang Gang” is consistent (*P* value is greater than 0.05). The first set of print works mainly reflects the artist's “affinity cold” emotion. The MSE values of the evaluation results are less than 0.01. That is, the color language analysis technology of print art based on GP-BP neural network can reflect the artist's emotion to a certain extent when analyzing the color language of the print.

## 1. Introduction

Printmaking plays an important role in art. With the progress of the times, people's spiritual and cultural aspects are developing in a diversified direction, and there are various ways of emotional expression [1]. The color language in print art can fully meet the needs of artists' emotional expression. Artists integrate their own subjective emotions into objective things. While describing objective things through color language in print art, they also express their own subjective emotions in color language. In other words, color language is an important medium for creators to express their inner feelings [2, 3]. The understanding of the color language of print art needs a certain degree of artistic accomplishment and the depth of knowledge related to print. For ordinary people, it is difficult to quickly have a basic understanding of the color of print language by themselves without a guide. Therefore, this paper proposes a printmaking art color language analysis technology based on GP-BP neural network aesthetic paradigm, which aims to provide some help for the viewers to understand the printmaking art language. Among them, the gradient boosting (GP) algorithm is a reinforcement learning algorithm, which combines several weak learning models in the form of iterating to minimize the loss function and then forms a strong learning model, which can improve the learning accuracy [4]. BP neural network belongs to error back propagation neural network, which is composed of input layer, hidden layer, and output layer, and is widely used [5]. In the process of research, GP algorithm is used to improve BP neural network algorithm, and GP-BP neural network is used to obtain the relationship between print color value and perceptual evaluation value, so as to carry out the language analysis of print art color.

RETRACTED

In recent years, more attention has been paid to the theoretical perception of art history, and there is a lack of investment in the research of art color. Strong et al. have discussed the relationship between color selection and visual perception, which provides a reference for understanding the color matching choice of Egyptian artists [6]. Laia et al. from the perspective of language, philosophy and specialty and others discussed the skills and connotation of painting art [7]. Lobatskaya et al. discussed in detail the division and organization of the space environment in the art museum with the painting object as the object and analyzed the reflection of the color matching and the trend of the contour line in the painting works on the works' emotion [8]. Malcolm et al. believed that landscape painting is a world of tranquility and natural beauty created by artists in space [9]. Hennen et al. conducted a nondestructive analysis on the paintings of Italian painter Carlo Saraceni through infrared reflection imaging and X-ray fluorescence spectroscopy and distinguished all the changes in the paintings through imaging examination, thus deepening the understanding of this work [10]. On the basis of fully understanding the painting color language, Rosario et al. have designed an interactive system, which can be applied to the painting of individual objects such as fruits, flowers, and leaves [11]. In order to detect the unauthorized use of copyright art painting, Hong et al. designed an object detector based on deep learning on the basis of analyzing the color language of painting art and combined with the color language to identify the art painting area [12].

Wei et al. used the gradient lifting algorithm to optimize the traditional machine learning algorithm and constructed the extreme gradient enhancement algorithm based on the optimal features of protein sequence. Compared with the traditional machine learning algorithm, the latter has higher recognition rate for type IV secretion effector [13]. Nutalapati et al. proposed the introduction of online gradient lifting algorithm when studying the online trajectory design problem in time-varying environment. The results show that the introduction of GP algorithm realizes the optimization of online trajectory with imprecise gradient feedback in spatiotemporal environment [14]. Flachot et al. used *K*-means clustering algorithm to classify the plaques in color images, and by changing the hue to measure the hue of the unit, they proposed a convolution neural network model based on hue [15]. Pdmf et al. have trained a detection convolution neural network using synthetic images. The detection results of real images show that the neural network can detect a variety of colors, which has a certain auxiliary role in color language analysis [16]. Han et al. proposed using convolution neural network to complete the fitting of bias color and real color, improve the camera's shooting quality of painting works, and ensure the authenticity of the color language of works [17]. Liu et al. proposed using BP neural network to segment retinal vessels in color fundus images, which shows that BP neural network has application value in color analysis [18].

RETRACTED

To sum up, in recent years, there are a lot of researches on artificial neural network, printmaking art, painting art, color analysis, and so on, but there is a lack of research on color language analysis of printmaking art through artificial neural network. Therefore, this paper proposes a color language analysis technology of print art based on GP-BP neural network aesthetic paradigm to help people quickly understand the emotions reflected in print art. The research process is shown in Figure 1.

## 2. Based on the GP-BP Neural Network Aesthetic Paradigm of Print Art Color Language Analysis Model Construction

### 2.1. Color Image Perception Evaluation Based on Semantic Difference Method

The traditional BP neural network adopts gradient descent method, but in the face of more complex objective function, the learning speed is not obvious enough, which reflects the low efficiency of the algorithm [19–22]. According to the gradient lifting method mentioned in previous studies, it is added to BP neural network, which solves the disadvantages of traditional BP neural network to a certain extent. The advantage of gradient lifting method is that it can perform well in the face of complex datasets with binary and continuous features. In this study, for the printmaking art language, we need to face the color difference and the analysis of the use of target color at the same time. Obviously, a simple neural network cannot be completed. Therefore, this study adds a gradient lifting algorithm based on the self-learning ability of BP neural network, which effectively improves the low efficiency of BP neural network.

RETRACTED

Color has three objective attributes, such as hue, lightness, and saturation. Human psychology of color belongs to the process of natural formation—from color perception to color association, then to color symbol and color perceptual intention. The color language of print art is based on color psychology, which is a way of transmitting certain information to the viewer through color [23, 24].

As can be seen from Figure 2, after the color of an object enters the human eye and is transmitted to the brain, it is recognized by the brain to classify the color and form the perception of color. The process of color perception is the process of causing human psychological reaction. After the visual organs are stimulated by the external color, it will form a series of synesthesia phenomena in the brain and finally form a comprehensive image, which is also the language of print art color [25].

As shown in Figure 3, when the brain receives a similar stimulus again, it will quickly associate with the memory of each other, complete the phenomenon of the thing, and complete the expression of the image of the thing with language, words and other ways, that is, the language communication with print art.

Figure 4 shows the percentage of perceptual image words and collocation samples, where *h* in HSB represents hue and *S* is saturation (1–100). The higher the saturation is, the higher the color is; *B* represents lightness (value is 1–100). The higher the lightness, the brighter the color [26, 27]. It can be seen that when 80% of the colors are warm, and 75% of the coordinate values meet *s* ≤ 60, *B* ≥ 80, it will show a friendly feeling to the print viewer. When 51% of the colors are inner white, 85% of the colors are warm, and 78% of the coordinate values satisfy *s* ≥ 80 and *B* ≥ 80, the print appreciators can realize the lively language conveyed by the print art.

As shown in Table 1, the combination of high saturation and high brightness cool tone with white inside print art color gives the viewer a sense of fashion, while the combination of black outside gives the viewer a modern texture. The design of low saturation and high brightness warm tone with inner white promotes the printmaking art to show a sense of affinity, while the design with outer black color shows a sense of luxury. When the low saturation and low brightness cold colors are combined with the outer white color design, the printmaking art shows a simple meaning as a whole, and when it is combined with the outer black color design, it shows a cold feeling.

RETRACTED

### 2.2. Analysis of Print Art Language Based on GP-BP Neural Network Aesthetic Paradigm

According to the relationship between color image vocabulary and collocation, after distinguishing the difference of color image perception in different print art, the paper uses GP-BP neural network to analyze the print art language. Gradient promotion (GP) algorithm combines weak prediction model to form strong prediction model [28]. When the number of weak classifiers is *M*, gradient upgrades to *m*, where *m* ∈ [0, *M*). The gradient lifting algorithm does not change the original prediction model *F*_*m*_(*x*). Instead, add predictors *h* to build a new prediction model in a new way *F*_*m*+1_(*x*) in the following equation:

(1) $$\begin{array}{c} F_{m+1}\left(x\right)=F_{m}\left(x\right)+h\left(x\right), \end{array}$$

where the residual error *h*(*x*) is a loss function (1/2)[*F*_*m*+1_(*x*) − *F*(*x*)]^2^. The negative gradient of the input variable is *x*, the output variable is *y*, and *F*_*m*+1_(*x*)=*F*_*m*_(*x*)+*h*(*x*)=*y*. Through joint probability *P*(*x*, *y*), the training set is assumed to be {*x*, *y*}_*i*=1_^*n*^. To minimize the loss function expectations of *L*(*y*, *F*(*x*)), it makes a special solution *F*^*∗*^(*x*).

(2) $$\begin{array}{c} F^{\wedge }\left(x\right)=\underset{F}{\arg\min}E_{x,y}\left[L\left(y,F\left(x\right)\right)\right], \end{array}$$

where *x* and *y* are input variables and output variables. *L*(*y*, *F*(*x*)) represents the loss function *F*. It refers to the prediction model. Set true value *y* after the weighting operation.

(3) $$\begin{array}{c} F^{\wedge }\left(x\right)=\sum_{i=1}^{n}\gamma_{i}h_{i}\left(x\right)+\text{const,} \end{array}$$

where const represents constant and training dataset (*x*_*i*_, *y*_*i*_), (*i*=1,2,…, *N*). *γ* represents the negative gradient direction of the loss function and *n* is the number of lifting steps.

(4) $$\begin{array}{c} F_{0}\left(x\right)=\underset{\gamma }{\arg\min}\sum_{i=1}^{n}L\left(y_{i},\gamma \right). \end{array}$$

Equation (4) is a constant function *F*_0_(*x*). The calculation formula of the model is expanded by greedy strategy. See the following formula for the extension process:

(5) $$\begin{array}{c} F_{m}\left(x\right)=F_{m-1}\left(x\right)+\underset{h\in H}{\arg\min}\sum_{i=1}^{n}L\left(y_{i},F_{m-1}\left(x_{i}\right)+h\left(x_{i}\right)\right), \end{array}$$

where *h* represents a predictor, and *h* ∈ *H*, *L*(*y*, *F*(*x*)) represents the loss function, *h*_*i*_(*x*) represents the base learner, and *F*_*m*−1_(*x*) indicates that the gradient is raised to *m* − 1. The prediction model is obtained at the same time. Considering the continuity of domain, the definition of *H* is the domain *R*. The above is a set of fractional functions, and at this time, the following formula can be obtained:

(6) $$\begin{array}{c} F_{m}\left(x\right)=F_{m-1}\left(x\right)+\gamma_{m}\sum_{i=1}^{n}\nabla F_{m-1}L\left(y_{i},F_{m-1}\left(x_{i}\right)\right), \end{array}$$

(7) $$\begin{array}{c} \gamma_{m}=\underset{\gamma }{\arg\min}\sum_{i=1}^{n}L\left(y_{i},F_{m-1}\left(x_{i}\right)-\gamma \frac{\partial L\left(y_{i},F_{m-1}\left(x_{i}\right)\right)}{\partial F_{m-1}\left(x_{i}\right)}\right). \end{array}$$

In equations (6) and (7), *γ* represents the negative gradient direction of the loss function and *F*_*m*−1_(*x*) indicates that the gradient is raised to the second level *m* − 1. The prediction model is obtained at the same time. When the definition field is discrete, the function set is *H* in this case and choose the closest loss function *L* candidate function of gradient *h*.

RETRACTED

As shown in Figure 5, the study adopts a three-layer BP neural network model, so that the number of input neurons and output neurons is *m* and *P* in turn, and the number of hidden layer neurons is *n*. At this time, the *m*th neuron in the input layer is represented by XM, and the *n*th neuron in the hidden layer and the *p*th neuron in the output layer are represented by Zn and YP in turn. The connection weights from the input layer to the hidden layer are represented by WMN, and the connection weights from the hidden layer to the output layer are represented by Wnp.

(8) $$\begin{array}{c} n<\sqrt{m+p}+a. \end{array}$$

Equation (8) is the number of neurons in the hidden layer *n*. Select the empirical formula for reference, where *m* indicates the number of input layer nodes, *p* indicates the number of output layer nodes, and *a* represents any constant of the interval (0, 10).

(9) $$\begin{array}{c} f\left(x\right)=\frac{1}{\left(1+e^{-x}\right)}. \end{array}$$

Equation (9) is a sigmoid-type nonlinear function acting on each neuron *f*(*x*). *x* is the value of the input function.

(10) $$\begin{array}{c} {\text{net}}_{k}=\sum_{j}\omega_{kj}O_{j}+\theta_{k}, \end{array}$$

(11) $$\begin{array}{c} O_{k}=f\left({\text{net}}_{k}\right). \end{array}$$

In formulas (10) and (11), *ω*_*kj*_ represents a neuron *U*_*k*_ to the upper layer of neurons, *U*_*j*_ represents the weight value of the connection between them, and *O*_*j*_ represents a neuron *U*_*j*_. When BP neural network is used as a weak learning model, the loss function is *ψ*(*y*, *f*)=(1/2) · (*y* − *f*(*x*))^2^, and the residual error is (*y* − *f*(*x*)) of which *f*(*x*). It is the fitting value of the model. The next BP neural network is trained along the direction of gradient descent, and then GP-BP neural network is realized.

(12) $$\begin{array}{c} \hat{f}\left(x\right)=f_{0}\left(x\right)+\sum_{i=1}^{M}\rho_{i}\cdot h\left(x,\theta_{i}\right). \end{array}$$

Formula (12) is the calculation formula of model fitting value of test data, where *ρ*_*i*_ represents the optimal reduced step size, weak learning model *h*(*x*, *θ*). The experimental program is run in MATLAB 2014a. When building a printmaking art color language analysis model based on GP-BP neural network, the color value and different printings are selected as the input layer, and the image evaluation value is taken as the output layer. After the training, the model is used for printmaking art color language analysis [29].

RETRACTED

As shown in Figure 6, firstly, according to the unique semantic differences of different colors, the perceptual evaluation of color image is carried out, and the relationship between perceptual image vocabulary and color matching of print art is found out. Secondly, through the gradient promotion (GP) method, the learning ability of BP neural network is enhanced and its loss function is reduced, and the GP-BP neural network model is constructed. Secondly, the color language analysis and evaluation model of print art based on GP-BP neural network model is constructed. Choose different print works, input the specific information of different print works, and finally output the image evaluation results of different print art color, which is the result of print art color language analysis.

## 3. The Result of Color Language Analysis of Print Art

### 3.1. Analysis of the Adjective Groups of Color Image in Print Art

Through questionnaire survey, the color image evaluation values of three types of prints, such as copper engraving, wood engraving, and hemp glue engraving, were obtained. The number of valid questionnaires was 70. Six image adjectives such as “heavy light,” “modern classical,” “lively steady,” “luxurious simple,” “soft masculine,” and “warm cold” are used as coordinate variables to draw the color image evaluation spatial distribution map of three types of prints, such as copper engraving, wood engraving, and hemp glue engraving.

As shown in Figure 7, 14 printmaking works with different contents are selected from each type of printmaking. According to the color types and their distribution on different printmaking works, the corresponding color image spatial evaluation distribution map is drawn. It can be seen that different types of engraving (copper engraving, wood engraving, and hemp glue engraving) have similar positions in the image distribution map, and there is no obvious distribution rule, which indicates that there is no obvious difference in color image perception among copper engraving, wood engraving, and hemp glue engraving. In order to verify whether the color images proposed in the study are different in different print types, the data were first tested for variance first, and then the data were analyzed by two-way ANOVA. When *P* < 0.05, the difference was statistically significant. The specific analysis results are shown in Figure 8.

RETRACTED

Figure 8 shows the two groups of image adjectives, such as “friendly cold” and “luxurious simple.” The corresponding *F* values are 5.939 and 3.713, respectively, and the *P* values are 0.008 and 0.038, respectively, which are less than 0.05. It shows that there are some differences in the perception and evaluation of two groups of color adjectives (color language expression) such as “warm cold” and “luxurious simple” in different types of print art works (copper print, wood print, and hemp glue print). The corresponding *F* values of four groups of image adjectives were 1.019, 1.227, 2.364, and 0.076, respectively, and the *P* values were 0.375, 0.310, 0.114, and 0.927, respectively, which were all greater than 0.05. It shows that there is no difference in the perception and evaluation of four groups of color adjectives (color language expression) in different types of prints (copper prints, wood prints, and hemp glue prints). The above results show that the color image adjectives can show the artistic language of different print types to a certain extent.

### 3.2. Analysis Results of Color Language Model in Print Art

In order to verify the practical application effect of the color language analysis technology of engraving art based on GP-BP neural network aesthetic paradigm proposed in this study, five pairs of completed engraving art works were randomly selected from three types of engraving art works, such as copper engraving, wood engraving, and hemp glue engraving. Through the color language analysis technology of print art based on GP-BP neural network aesthetic paradigm, this paper analyzes the five print art works, and the specific analysis results are shown in Figure 9.

It can be seen from Figure 9 that the emotional evaluation value of the adjective group of “friendly cold” color image expressed in the first print art work is the highest, reaching 0.9563. The second is the “luxurious simple” color image adjective with the perceptual evaluation value of 0.1609, and the color image adjective with the smallest perceptual evaluation value is “steady lively.” The above results show that the color language of the first printmaking works selected in this study mainly conveys the “friendly cold” emotion to the viewers. In the second print, the perceptual evaluation value of “friendly cold” color image adjective group is 0.9995, the perceptual evaluation value of “luxurious simple” color image adjective group is 0.8694, and the perceptual evaluation value of “leisure modern” color image adjective group is 0.9927. It shows that the color language of the second print works mainly conveys emotions to the outside world, including “friendly cold,” “luxurious simple,” “leisure modern,” and so on. In the third and fourth prints, the adjectives of color image with the highest perceptual evaluation value are “retro trendy,” which shows that the two prints mainly show the outside world the classification of retro trendy through color. In addition, the adjective of color image in the fourth print is “leisure modern,” and the perceptual evaluation value is 0.6275.

RETRACTED

In the experiment, the color language expression of the selected five prints was analyzed by questionnaire survey method, and 126 valid questionnaires were collected. The questionnaire was statistically analyzed, and the subjective evaluation of different human individuals on the color language expression of the five prints was counted. See Figure 10 for details.

Figure 10 shows that, in the evaluation of the color language expression content of the first print art works, the adjectives of color image are “friendly cold,” “luxurious simple,” “retro trendy,” “leisure modern,” and “steady lively,” and the corresponding subjective perceptual evaluation values are 0.9672, 0.1500, 0.0384, 0.0029, and 0.0007, respectively. In the evaluation of color language expression content of the second print, the adjectives of color image are “friendly cold,” “luxury simple,” “retro trendy,” “leisure modern,” and “steady lively,” and the corresponding subjective perceptual evaluation values are 1.0000, 0.8667, 0.3003, 0.9767, and 0.0002, respectively. In the evaluation of color language expression of the third print, the adjectives of color image are “affinity cold,” “luxury simple,” “retro trendy,” “leisure modern,” and “steadiness liveliness,” and the corresponding subjective perceptual evaluation values are 0.0533, 0.0003, 0.6378, 0.1356, and 0.0002, respectively. In the evaluation of color language expression of the fourth print, the adjectives of color image are “friendly cold,” “luxurious simple,” “retro trendy,” “leisure modern,” and “steady lively,” and the corresponding subjective perceptual evaluation values are 0.0743, 0.0041, 0.9229, 0.6386, and 0.0040, respectively. This paper compares the subjective evaluation of color language expression of print art works with the analysis results of color language of print art based on GP-BP neural network aesthetic paradigm and verifies the feasibility of the proposed analysis technology of color language of print art according to the comparison results. The specific comparison results are shown in Figure 11.

RETRACTED

As can be seen from Figure 10, the differences between the subjective evaluation results and the network algorithm evaluation results are 0.0109, 0.0005, 0.0015, 0.0036, and 0.0033, respectively, for the perceptual evaluation value of the color image adjective “affinity cold.” On the perceptual evaluation value of “steady and lively,” the differences of the two evaluation methods are 0.0004, 0.0001, 0.0001, 0.0001, and 00001, respectively. When the standard deviation of all the data is verified, the corresponding MSE values are less than 0.01, which indicates that the results are valid. In other words, the color language analysis technology of print art based on GP-BP neural network aesthetic paradigm proposed in this study is feasible in the analysis of print color language.

## 4. Conclusion

Print art color language reflects the artist's subjective feelings; different color collocation contains different color language. In order to help viewers quickly understand the main emotions of the artists in the print art works, this paper designs a print art color language analysis technology based on GP-BP neural network aesthetic paradigm on the basis of extracting the common color image adjectives of print art, and selects five different print art works. The results show that the extracted color image adjectives can adapt to the color language expression of different types of engraving, such as copper engraving, wood engraving, and hemp and glue engraving. On the three kinds of material prints, the expression effect of image adjectives “leisure modern,” “retro trendy,” “lively steady,” and “soft masculine” is consistent (*F* = 1.019, 1.227, 2.364, and 0.076; *P*=0.375,  0.310,  0.114,  and 0.927). In the first print, the color language mainly expresses “affinity cold” emotion, and the corresponding perceptual evaluation value is 0.9563. The second print mainly expresses “affinity cold” (0.9995), “luxury simple” (0.8694), and “leisure modern” (0.9927) emotions. The third print mainly expresses “retro trendy” emotion. The fourth print mainly expresses the emotion of “retro trendy” and “leisure modern.” The MSE values of subjective evaluation results and network evaluation results were less than 0.01. To sum up, the color language analysis technology of print art based on GP-BP neural network is feasible. Although the method proposed in the research can well realize the artistic language analysis in printmaking, it can still be seen that the proposed method also has corresponding shortcomings. It is undeniable that the contour of color will affect the effect of printmaking language expression, and how to reduce the influence of contour will be the direction of further research.

RETRACTED

## Figures and Tables

**Figure 1:** Research process.

**Figure 2:** Color perception.

**Figure 3:** Image formation and expression concept map.

**Figure 4:** Statistical chart of perceptual image vocabulary and collocation samples.

**Figure 5:** Schematic diagram of 3-layer BP neural network.

**Figure 6:** Flowchart of color language analysis in print art.

**Figure 7:** Spatial distribution of color image of three types of prints.

**Figure 8:** Two-way ANOVA of image adjective pairs of different products.

**Figure 9:** The analysis results of color language of print art based on GP-BP neural network aesthetic paradigm. (a) The first print, (b) the second print, (c) the third print, (d) the fourth print, and (e) the fifth print.

**Figure 10:** Subjective evaluation results of 5 prints.

**Figure 11:** Comparison of subjective evaluation results and technical evaluation results based on GP-BP. *Note*. MSE is the mark difference, which mainly indicates the accuracy of measurement. When MSE is less than 0.01, the result is valid.

**Table 1:** The relationship between perceptual image words and collocation samples.

Project	Inner white color matching	Inner black color matching	Exterior black color matching	Exterior white color matching
High saturation, high brightness, and cool tone	New trend	New trend	Modern	Leisure time
High saturation, high brightness, and warm tone	Lively	Lively	Luxury	Affinity
Low saturation, high brightness, and cold tone	Simple	Simple	Modern	Leisure time
Low saturation, high brightness, and warm tone	Affinity	Affinity	Luxury	Affinity
High saturation, low brightness, and cool tone	Simple	Steady	Modern	Simple
High saturation, low brightness, and warm tone	Retro	Steady	Grim	Retro
Low saturation, low brightness, and cool tone	Simple	Simple	Grim	Simple
Low saturation, low brightness, and warm tone	Retro	Retro	Grim	Retro

## Data Availability

The data used to support the findings of this study are available from the corresponding author upon request.
